# K-Means Segmentation of Underwater Image Based on Improved Manta Ray Algorithm

**DOI:** 10.1155/2022/4587880

**Published:** 2022-03-16

**Authors:** Donglin Zhu, Linpeng Xie, Changjun Zhou

**Affiliations:** ^1^College of Mathematics and Computer Science, Zhejiang Normal University, Jinhua 321004, China; ^2^School of Information Engineering, Jiangxi University of Science and Technology, Ganzhou, Jiangxi 341000, China

## Abstract

Image segmentation plays an important role in daily life. The traditional K-means image segmentation has the shortcomings of randomness and is easy to fall into local optimum, which greatly reduces the quality of segmentation. To improve these phenomena, a K-means image segmentation method based on improved manta ray foraging optimization (IMRFO) is proposed. IMRFO uses Lévy flight to improve the flexibility of individual manta rays and then puts forward a random walk learning that prevents the algorithm from falling into the local optimal state. Finally, the learning idea of particle swarm optimization is introduced to enhance the convergence accuracy of the algorithm, which effectively improves the global and local optimization ability of the algorithm simultaneously. With the probability that K-means will fall into local optimum reducing, the optimized K-means hold stronger stability. In the 12 standard test functions, 7 basic algorithms and 4 variant algorithms are compared with IMRFO. The results of the optimization index and statistical test show that IMRFO has better optimization ability. Eight underwater images were selected for the experiment and compared with 11 algorithms. The results show that PSNR, SSIM, and FSIM of IMRFO in each image are better. Meanwhile, the optimized K-means image segmentation performance is better.

## 1. Introduction

In recent years, image segmentation has attracted much attention and research by researchers. It is of great significance to the future image processing field. As a key step of image processing, image segmentation plays an important role in extracting objects of interest from images. At present, it has important research value in medicine, agriculture, ocean, and other fields. Image segmentation can be divided into four categories: threshold segmentation, region segmentation, edge segmentation, and segmentation methods based on specific theories. The clustering algorithm is a typical unsupervised learning algorithm. It uses the idea of clustering differentiation to solve the problem. The way to solve the problem is simple and easy to understand. It has been successfully applied in many fields [1]. Cluster image segmentation has also been successfully studied. K-means is the most common and easiest clustering method among them, but K-means has the disadvantage of large randomness and easily fall into local optimum, which makes it impossible to control the cluster center reasonably. Swarm intelligence algorithms is an algorithm with global optimization performance and strong versatility that is suitable for parallel processing. This type of algorithm can find the optimal solution or approximate the optimal solution within a certain period of time. [2] Intelligent optimization algorithm opens up a new way for image segmentation. In terms of clustering segmentation, Hrosik *R* C and others improved the K-means clustering algorithm based on the firefly algorithm, which could achieve better segmentation average error, peak signal-to-noise ratio, and structural similarity index on medical images; [3] Li *h* and others proposed a k-means clustering algorithm based on dynamic particle swarm optimization (DPSO), which had better visual effect than traditional K-means clustering in image segmentation and obvious advantages in improving image segmentation quality and efficiency; [4] Shubham and others applied gray wolf optimizer (GWO) [5] to the segmentation of satellite images; [6] Therefore, an intelligent optimization algorithm is of great significance in the field of image segmentation.

With the rapid development of swarm intelligence algorithms, a variety of new algorithms are emerging. In addition to the algorithms mentioned above, there are other algorithms as follows: monarch butterfly optimization (MBO) [7], elephant herding optimization (EHO) [8], moth search (MS) algorithm [9], Harris hawks optimization (HHO) [10], etc. Manta ray foraging optimization (MRFO) is a new swarm intelligence optimization algorithm proposed in 2020. With excellent searchability, fewer parameters, simple model and easily understood, it is better than particle swarm optimization (PSO) [11, 12], genetic algorithm (GA) [13, 14], Differential Evolution (DE) [15, 16], Cuckoo Search (CS) [17], gravitational search algorithm (GSA) [18], and ABC [19] in some function optimization [20], and it has been successfully applied to solar energy [21, 22], ECG [23], generator [24, 25], power system [26], cogeneration energy system [27], geophysical inversion problem [28], directional overcurrent relay [29], feature selection [30], hybrid energy system [31], and sewage treatment [32]. Although MRFO has good optimization ability, it still has its own defects. In complex problems, the search ability is limited and the diversity of the population can not be guaranteed. The main reason is that the individual searches orderly, highly dependently, and inflexibly.

At present, researchers have noticed this point and carried out successive studies, such as Mohamed Abd Elaziz, who combines fractional calculus with MRFO to correct the direction of manta ray movement. This algorithm has been verified by CEC 2017 test function and is applied to image segmentation problems with good feasibility [33]. Mohamed H. Hassan combines a gradient optimizer with MRFO to reduce the probability that the algorithm will fall into a local optimum, which has a good effect in single-objective and multiobjective economic emission scheduling [34]. Haitao Xu uses adaptive weighting and chaos to improve MRFO, so as to efficiently handle thermodynamic problems [35]. Essam H. Houssein uses reverse learning to initialize the population so as to increase the diversity of the population and apply it to the threshold image segmentation problem with good segmentation quality [36]. Bibekananda Jena adds an attack capability to MRFO, which allows it to jump out of local optimization and find a globally optimal solution. It is then applied to the image segmentation problem of 3D Tsallis [37]. Mihailo Micev fuses Simulate Anneal (SA) with MRFO and applies it to the Proportional Integral Derivative (PID) controller. The fused algorithm is superior to other algorithms [38]. In addition, Serdar and others adopt opposition-based learning and SA to improve the convergence effect of MRFO. It has better control performance when applied to fractional order proportional integral derivative (FOPID) controller [39]. Although the currently proposed variants of MRFO have achieved some results, the following problems still exist:

1. Most scholars use the fusion of other algorithms to improve the search ability, but this will bring higher time complexity, and the algorithm after fusion may not be able to complement each other so as to present perfect results.
2. Reverse learning can only solve inversely in a certain space, but in complex high-dimensional situations, there are fewer individual optimization methods, and they cannot jump out of the local optimal state perfectly.
3. In the optimization process, the above algorithm cannot completely balance the local search and global search capabilities, which results in insufficient convergence accuracy of the algorithm.

Based on the above analysis, this paper presents an improved algorithm for manta rays, which uses random walk learning to make individuals wander randomly in space, to increase the diversity of the population, and avoid premature convergence of the algorithm, and then we use Lévy flight for long-distance and short-distance searches to balance the local and global searches of the algorithm. Finally, the learning idea of particle swarm is introduced. Two learning factors are used to improve the convergence accuracy of the algorithm 12 functions are used to verify the validity and feasibility of IMRFO. Then eight underwater image datasets are used in K-means image segmentation. The results show that IMRFO has better generalization ability and better segmentation quality.

The innovations and contributions of this paper are as follows:

- A random walk learning algorithm is designed to increase the diversity of the population and reduce the probability of the algorithm falling into local optimization to a certain extent.
- Lévy flight and learning factors are introduced to balance the searchability of the algorithm, which makes the algorithm have a good convergence effect.
- In 12 standard test functions, IMRFO is compared with 7 other algorithms to show its superiority and feasibility. Next, two statistical tests are used to emphasize the optimization performance of the algorithm. It is compared with the recently proposed variants of the algorithm. Finally, ablation experiments were performed, all the results show that IMRFO has a good search ability.
- IMRFO is applied to K-means underwater image segmentation. The results of 11 algorithms show that IMRFO performs well.

The structure of this paper is as follows: Section 2 introduces the basic MRFO algorithm, Section 3 introduces the improved IMRFO algorithm and related analysis.  Section 4 describes the process of IMRFO optimizing K-means image segmentation.  Section 5 tests the performance of IMRFO and compares the related algorithms.  Section 6 describes and analyses the performance of each algorithm in K-means image segmentation.  Section 7 summarizes the experimental results of this paper. The last section expresses the advantages and disadvantages of IMRFO and future research directions.

## 2. Manta Ray Foraging Optimization

Manta rays feed on plankton, which are mainly water microfauna. When feeding, they suck water and prey into their mouths with angular head leaves. They then filter prey out of the water through improved rabbles. Individuals of the manta rays work together to find the best food. Inspired by the behavior of the manta rays, the algorithm is divided into chain feeding, spiral-feeding, and somersault foraging. There are three stages of spiral and empty foraging.

### 2.1. Chain Feeding

At this stage, the manta ray population will be arranged in an ordered chain to collaborate in feeding, which will maximize the amount of plankton in the pocket. The mathematical model of the chain feeding process can be expressed as follows:

(1) $$\begin{array}{c} x_{i}^{d}\left(t+1\right)=\left\{\begin{array}{cc} x_{i}^{d}\left(t\right)+r\cdot \left(x_{\text{best}}^{d}\left(t\right)-x_{i}^{d}\left(t\right)\right)+\alpha \cdot \left(x_{\text{best}}^{d}\left(t\right)-x_{i}^{d}\left(t\right)\right), & i=1,\\ x_{i}^{d}\left(t\right)+r\cdot \left(x_{i-1}^{d}\left(t\right)-x_{i}^{d}\left(t\right)\right)+\alpha \cdot \left(x_{\text{best}}^{d}\left(t\right)-x_{i}^{d}\left(t\right)\right), & i=2,3,\ldots ,N. \end{array}\right. \end{array}$$

In formula (1), *x*_*i*_^*d*^(*t*) denotes the d-dimensional information of the location of the first manta ray in generation *t*. *R* is a random number that obeys a uniform distribution of [0,1]. $\alpha =2\cdot r\cdot \sqrt{\left|\log\left(r\right)\right|}$ is the weight factor, *x*_best_^*d*^(*t*) is the d-dimensional information of the best location found so far The manta ray at position *i* depends on the manta ray at position i-1 and the best food position found so far. *N* represents the population number. The update of the first manta ray depends on the optimal location.

### 2.2. Spiral Feeding

When a manta ray finds a good food source in a certain space, each individual approaches a manta ray in front of it, in addition to spirally moving toward the food. The spiral-feeding process can be represented by the following mathematical model:

(2) $$\begin{array}{c} x_{i}^{d}\left(t+1\right)=\left\{\begin{array}{cc} x_{best}^{d}\left(t\right)+r\cdot \left(x_{best}^{d}\left(t\right)-x_{i}^{d}\left(t\right)\right)+\beta \cdot \left(x_{best}^{d}\left(t\right)-x_{i}^{d}\left(t\right)\right), & \;i=1,\\ x_{best}^{d}\left(t\right)+r\cdot \left(x_{i-1}^{d}\left(t\right)-x_{i}^{d}\left(t\right)\right)+\beta \cdot \left(x_{best}^{d}\left(t\right)-x_{i}^{d}\left(t\right)\right), & i=2,3,\ldots ,N. \end{array}\right. \end{array}$$

where *β*=2*e*^*r*_1_(*T* − *t*+1)/*T*^ · sin(2*πr*_1_), a weight factor representing the spiral motion, *T* being the largest number of iterations, *r* being the rotation factor and obeying [0,1] uniform random numbers. In addition, in order to improve the efficiency of population foraging, MRFO randomly generates a new location during the optimization process and then performs a spiral search at that location. Its mathematical model is as follows:

(3) $$\begin{array}{c} x_{i}^{d}\left(t+1\right)=\left\{\begin{array}{cc} x_{\text{rand}}^{d}\left(t\right)+r\cdot \left(x_{\text{best}}^{d}\left(t\right)-x_{i}^{d}\left(t\right)\right)+\beta \cdot \left(x_{\text{best}}^{d}\left(t\right)-x_{i}^{d}\left(t\right)\right), & i=1,\\ x_{\text{rand}}^{d}\left(t\right)+r\cdot \left(x_{i-1}^{d}\left(t\right)-x_{i}^{d}\left(t\right)\right)+\beta \cdot \left(x_{\text{best}}^{d}\left(t\right)-x_{i}^{d}\left(t\right)\right), & i=2,3,\ldots ,N. \end{array}\right. \end{array}$$

*x*_rand_^*d*^(*t*) represents a new location in space.

### 2.3. Somersault Foraging

When a certain manta ray finds a food source, its position can be regarded as an axis. Each manta ray tends to wander around the axis and flip to a new location. Its mathematical model is as follows:

(4) $$\begin{array}{c} \begin{array}{c} x_{i}^{d}\left(t+1\right)=x_{i}^{d}\left(t\right)+S\cdot \left(r_{2}\cdot x_{\text{best}}^{d}\left(t\right)-r_{3}\cdot x_{i}^{d}\left(t\right)\right),i=1,2,\ldots ,N \end{array}. \end{array}$$

*S* is the flip factor, which determines the flip distance. *R*_2_ and *r*_3_ are two random numbers that are uniformly distributed [0,1]. As *S* values vary, individual mantas flip to locations in search space that are symmetrical to the optimal solution at their current location.

## 3. Improved Manta Ray Foraging Optimization

From the above formulas, it can be seen that more communication between individuals and orderly work can improve the searchability of the algorithm and perform a wide-ranging search. On the one hand, the lack of initiative of individuals in the population limits their ability to develop. On the other hand, updates within the population are related to the best location. When encountering high-dimensional complex problems, the change of the optimal position is similar, which results in less change in the two updates before and after the algorithm, which limits the algorithm's optimization ability. Therefore, a flexible change strategy is needed to improve the development ability and local convergence effect of the algorithm. This paper uses the Lévy flight strategy to improve individual blindness search, and random walk learning is used to prevent the algorithm from falling into a local state and the learning idea of particle swarm to improve the search accuracy of the algorithm.

### 3.1. Why Each Modification Has Been Proposed?

MRFO is based on a group of animals collaborating in feeding, which results in fewer optimization methods and a lack of flexibility and fineness. Therefore, individual initiative is required to increase the diversity of the population in order to find high-quality solutions in space.

Therefore, this paper analyses and solves the defects of the algorithm from the following three points. Firstly, it is necessary to make the population individuals better distribute the whole space so as to develop the vision of the algorithm and improve the global search ability of the algorithm. Lévy flight is a classical strategy, which can fly in a given space in the way of alternating long and short distances. It has been used by most scholars to improve the search ability of the algorithm. Secondly, some individuals need to be independent and never be limited by group characteristics. Random walk learning is an uncertain way of walking. The traditional random walk can only be carried out in local areas. However, the random walk learning designed in this paper can make large location differences between different individuals and improve the population diversity of the algorithm. Finally, information sharing among individuals is needed to improve the local search ability of the algorithm and find high-quality solutions. The learning factor is derived from the particle swarm optimization algorithm, which is used to speed up the information exchange of the population, prevent the early invalid search, improve the local search ability of the algorithm, and improve the accuracy of the solution to a certain extent.

### 3.2. Lévy Flight Strategy

When manta ray individuals perform chain search, all individuals follow the population to search, which leads to the lack of flexibility of the algorithm and can not perform a better search range. Therefore, the Lévy flight strategy [40, 41] is introduced to enable individuals to search long and short distances, increase the diversity of the population, and enable individuals to fully diffuse into the whole space. The location update format for joining Lévy flight strategy is as follows:

(5) $$\begin{array}{c} x_{i}^{\prime }\left(t\right)=x_{i}\left(t\right)+l⊕\text{levy}\left(\lambda \right). \end{array}$$

In formula (8), x_i_(t) represents the position of the i-th individual in the t-th iteration, ⊕ is an arithmetic symbol representing point-to-point multiplication. l = 0.01(x_i_(t)-x_p_) denotes a step length control parameter, x_p_ represents the position of the best individual in the population.

Lévy flight formula is as follows [42]:

(6) $$\begin{array}{c} \begin{array}{c} \text{Levy}\left(x\right)=0.01\times \frac{r_{4}\times \sigma }{{\left|r_{5}\right|}^{\left(1/\xi \right)}} \end{array}. \end{array}$$

where *r*_4_ and *r*_5_ are random numbers within the range of [0,1], *ξ*. The general value is 1.5. *σ* is calculated as follows:

(7) $$\begin{array}{c} \sigma ={\left(\frac{\Gamma \left(1+\xi \right)\times \sin\left(\pi \xi /2\right)}{\Gamma \left(1+\xi /2\right)\times \xi \times 2^{\left(\xi -1/2\right)}}\right)}^{\left(1/\xi \right)}. \end{array}$$

where Γ(*x*)=(*x* − 1)!, the schematic diagram of Lévy flight is shown in Figure 1. Lévy flight can search long and short distances in a certain space and balance the global and local search of the algorithm.

### 3.3. Random Walk Learning

In the optimization process, MRFO has the probability of falling into the local optimum, which makes the current optimum individual unreliable, so it is necessary to disperse all the individuals to find a better solution. Unlike random walks, the learning factors at the best and worst locations are introduced to make individual escape directional and reduce unreasonable walk. The specific mathematical model of RWL is as follows:

(8) $$\begin{array}{c} x_{i,j}^{t+1}=x_{\text{best}}^{t}+\left(\frac{2}{1+t/M\cdot \sin\left(\pi /2\cdot r\right)}-1\right)\cdot e^{\left(-\frac{t}{M}\right)\cdot \left(x_{i,j}^{t}-x_{\text{worst}}^{t}\right)}+\left(c_{1}\cdot x_{\text{best}}^{t}-c_{2}\cdot X_{i,j}^{t}\right). \end{array}$$

In formula (8), ((2/1+*t*/*M*.sin(*π*/2.*r*)) − 1) is the sinusoidal random factor that uses the mathematical properties of the sinusoidal function to fluctuate toward the optimal solution and continuously adjusts the step size based on the worst position of the current population so that the search path can span the entire solution space. *M* is the maximum number of iterations, and *c*_*1*_ and *c*_*2*_ represent two learning factors, random numbers that obey a normal distribution. *e*^(−*t*/*M*).(*x*_*i*,*j*_^*t*^ − *x*_worst_^*t*^)^ is the control step, (*c*_1_.*x*_best_^*t*^ − *c*_2_.*X*_*i*,*j*_^*t*^) is the direction of control. As shown in Figure 2(a), (a) is the distribution of individuals without introducing RWL, (b) introduces the individual distribution of RWL; we can see that the introduction of RWL enables individuals to master global information, makes the individual distribution more even, and finds the global optimal solution.

### 3.4. PSO Algorithm Learning Ideas

There are two learning factors in PSO to develop local solutions, which can effectively improve the convergence accuracy of the algorithm. Therefore, the formula of introducing two learning factors is as follows:

(9) $$\begin{array}{c} x_{i,j}^{t+1}=b_{1}\cdot x_{i,j}^{t}+b_{2}\cdot \text{rand}\left(1\right)\cdot \left(\text{Best}X-x_{i,j}^{t}\right). \end{array}$$

*b*_*1*_, *b*_*2*_ are two learning factors, and *BestX* is the optimal position of the current population. As can be seen from the formula, this strategy exploits individuals between the current one and the optimal one to enhance the local search of the algorithm.

### 3.5. Improved Manta Ray Foraging Optimization

To improve the local search capability of MRFO and reduce the probability of falling into local optimum, an improved manta ray algorithm is presented in this paper. The algorithm uses random walk learning to prevent the algorithm from falling into the local state after each iteration and to improve the global search ability of the algorithm. Then, the Lévy flight mechanism is combined to improve the blindness of the manta ray algorithm and to balance the searchability of the algorithm. Using two learning factors of particle swarm optimization to improve the search accuracy ultimately makes the algorithm improve effectively both in local and global aspects. The specific pseudocode is shown in Algorithm 1.

## 4. K-Means Image Segmentation Based on IMRFO

The principle of the traditional K-means algorithm is to select K cluster centers randomly, so the way to select them is uncertain, resulting in large differences in the final results and easy to fall into local optimum. Therefore, it is necessary to select an appropriate initial cluster center. Intelligent optimization algorithm has been successfully applied to K-means to improve its randomness and the defect of falling into local optimum. The improved manta ray foraging optimization optimizes K-means so that the initial cluster centers are well controlled. The objective function is as follows:

(10) $$\begin{array}{c} f=\overset{n}{\underset{i=1}{\sum }}\overset{m}{\underset{j=1}{\sum }}{\left|X_{i}-Y_{i}\right|}^{2}. \end{array}$$

*X*_*i*_ is a pixel gray value of the image and *Y*_*i*_ is the J-th clustering center. The optimal initial number of clustering centers is obtained by IMRFO to minimize the fitness value of the objective function.

K-means image segmentation based on IMRFO is mainly divided into two parts:

1. Use the global search capabilities of IMRFO to find the best initial cluster center in the image point set
2. The initial cluster centers of the IMRFO output are segmented in the K-means algorithm

The specific flow chart is shown in Figure 3.

## 5. Performance Analysis and Test

### 5.1. Performance Test

To verify the effectiveness and feasibility of IMRFO, 12 benchmark functions [43, 44] are selected to verify its function optimization ability. The specific test function information is shown in Table 1. F1-6 is a unimodal function, F7-11 is a complex multimodal function, and F12 is a fixed-dimensional function. In addition, F1-11 is tested in different dimensions to verify the optimization ability of the algorithm in high-dimensional cases. To prove that IMRFO is competitive, seven algorithms including MRFO, Honey Badger Algorithm (HBA) [45], GWO, PSO, Whale Optimization Algorithm (WOA) [46], Learning Based Optimization (TLBO) [47], and Flower Pollution Algorithm (FPA) [48] are compared. The new cluster intelligence algorithm was proposed by HBA in 2021, while other algorithms are classical ones that have been extensively studied. The number of iterations and population of each algorithm are 500 and 100. In HBA, *O* = 6, *C* = 2; In FPA, the selection probability *p* = 0.8. B_1_ and *b*_2_ in IMRFO are 0.2 and 0.8, respectively. The experimental environment is Windows 10 64 bit; the software is matlab2019b; the memory is 16 GB; the processor is Intel(R) Core (TM) i5-10200H CPU @ 2.40 GHz. The average, optimal value, and standard deviation of the results of each algorithm for 30 runs are calculated. If IMRFO is the optimal value, the font is bolded. The optimization results of each algorithm are calculated as shown in Table 2-3.

On the one hand, from Table 2 and Table 3, we can see that IMRFO has obvious advantages in searching ability, and the results are better than other algorithms in each function. The increase of dimension does not reduce the searching ability of IMRFO. On the other hand, among these functions, F1, F6, F8-10, F12, MRFO itself has a good optimization effect and can find the theoretical optimal value, IMRFO also has the same optimization effect, so it can be seen that IMRFO does not weaken the original algorithm's optimization ability. Overall, IMRFO has been effectively improved in stability and accuracy. It can be seen that the introduction of multiple strategies improves the algorithm's optimization ability and reduces the probability of entering a local optimum.

### 5.2. Statistical Test

To verify whether IMRFO and the other seven algorithms have significant differences in global optimization, the 30-dimension results of each algorithm are tested. The Wilcoxon rank-sum test is used to find the differences between the two algorithms. Assume H0 : The two algorithms have the same performance. H1 : There is an obvious difference between the two algorithms. Use the *P*-value of the test results to measure the differences between the two algorithms. When *P* < 0.05, reject H0. It shows that there is a significant difference between the two algorithms. When *P* > 0.05, H0 is accepted, indicating that the two algorithms have the same global optimization performance. To clearly see the differences between these algorithms, we utilize N/A to represent the values of *P* > 0.05. The Wilcoxon test results are shown in Table 4. At the same time, in order to better show the comprehensive optimization ability of IMRFO in the whole test function, the average and variance of each algorithm are Friedman test [49], and the final ranking is calculated to measure the universality of the algorithm in the 12 test functions. The test results are shown in Table 5.

From Table 4, it can be seen that IMRFO differs significantly from other algorithms. In some functions, MRFO itself has better searching ability, so the difference is not obvious. From Table 5, IMRFO ranks best in the search results of each function, which also indicates that it has a good universality.

### 5.3. Comparison with Variants of the Algorithm

To further show the effectiveness and innovation of IMRFO, this paper compares IMRFO with multistrategy serial cuckoo search algorithm (MSSCS) [50], firefly algorithm with courtship learning (FACL) [51], self-adaptive cuckoo search (SACS) [52], and CSsin [53] proposed in recent years. These four algorithms are variants of classical algorithms and have been validated in the CEC test set. The specific parameters of each algorithm are set as follows: In MSCS algorithm, *α* = 0.01,* β* = 1.5, *P*_*a*_ = 0.25, *C* = 0.2, *PA*_*max*_ = 0.35, *PA*_*min*_ = 0.25; in CSsin algorithm, *P*_max_ = 0.75, *P*_max_ = 0.25, *freq* = 0.5; in FACL, *α* = 0.01,* β*_min_ = 0.2,* β* = 1, *γ* = 1. The number of populations and the number of iterations for each algorithm are shown above. Similarly, when IMRFO is the optimal value, font bolding will be applied. The results of each algorithm are shown in Table 6.

From Table 6, it is clear that IMRFO is the best value in F1-4, F6, F9-12, which shows that IMRFO is better than these algorithms in the optimization of these functions. Secondly, the variants of CS have better optimization results, especially in F5 and F7, which have higher accuracy. FACL, as the worst one, has poor optimization results but good stability. Generally speaking, IMRFO has some advantages in function optimization, which verifies the effectiveness and innovation of the algorithm.

### 5.4. Convergence Analysis

In order to clearly see the optimization and convergence effect of each algorithm in each function, the average convergence diagram of each algorithm is given as shown in Figure 4.

From Figure 4, it can be seen that IMRFO has a good convergence effect and can find the most accurate solution quickly, especially in the functions of F1-4, F6, F11. It can be seen that the flexible search mechanism enables the algorithm to find the best solution quickly in the optimization process.

### 5.5. Ablation Experiment

In order to verify the validity and feasibility of the three combinations of strategies, the combinations of strategies are experimented with to find the better one. In this paper, the algorithm of combining Lévy flight with GWL is recorded as MRFO-I, the algorithm of combining Lévy flight with PSO learning thought strategy is recorded as MRFO-II, while the algorithm of combining PSO thought with GWL is recorded as MRFO-III. Besides, the algorithm using Lévy flight alone is recorded as MRFO-IV, the algorithm using GWL alone as MRFO-V, and the algorithm utilizing PSO alone as MRFO-VI. The experimental parameters are consistent with those above. The test function dimension is 30. If IMRFO is the optimal value, the font is bolded. The experimental results are shown in Table 7.

As can be seen from Table 7, IMRFO is the best performer of all variants, and the criteria on each function are the best. IMRFO search accuracy is better than other algorithms and the difference is significant especially in F2, F4, F11. Therefore, it can be seen that the integration of multiple strategies is important, and the validity and feasibility of IMRFO are verified.

### 5.6. Time Complexity Analysis

Time complexity is an important measure of an algorithm. In order to show an effective improvement, it is necessary to balance the searchability and time complexity of the algorithm. The basic MRFO consists of only three phases, chain feeding, spiral feeding, and empty feeding, where chain feeding and spiral feeding are in the same cycle. Set the population number to *N* and the maximum number of iterations to *T*. The dimension is *D*, so the time complexity of MRFO can be summarized as follows. Macroscopically, the time complexity of swarm intelligence algorithms is the product of population number, iteration number, and dimension. Therefore, the time complexity of IMRFO is O (TND), just like other algorithms.

Microscopically, MRFO can be calculated as follows:

(11) $$\begin{array}{c} O\left(\text{IMRFO}\right)=O\left(T\left(O\left(\text{cyclone foraging}+\text{ chain foraging}\right)+O\left(\text{somersault foraging}\right)\right)\right)\\ =O\left(T\left(ND+ND\right)\right)=O\left(TND\right). \end{array}$$

Set the calculation time of introducing RWL to be t1, the calculation time of introducing Lévy flight to be *t*_2_, the calculation time of using two learning factors to be *t*_3_, and the other calculations are ignored.

IMRFO can be summarized as follows:

(12) $$\begin{array}{c} O\left(\text{MRFO}\right)=O\left(T\left(O\left(\text{cyclone foraging}+\text{ chain foraging}\right)+O\left(t1\right)+O\left(\text{somersault foraging}\right)+O\left(t_{2}\right)+O\left(t_{3}\right)\right)\right)\\ =O\left(TND\right). \end{array}$$

Therefore, it can be seen that the time complexity of IMRFO has not changed fundamentally. A small increase in the number of iterations can be ignored. These increases will be of great significance if the optimization capability of the algorithm is effectively improved.

## 6. Image Segmentation Experiments

At present, image processing has been applied in many fields, and the image on land has been well developed, but it still has research value in underwater images. So in order to show the research value, eight underwater images are selected as test images. From the literature [54], select PSO, DPSO, sparrow search algorithm (SSA) [55], Modified sparrow search algorithm (MSSA) [56], ABC, MRFO, WOA, TLBO, FPA, IMRFO 9 algorithms optimize K-means algorithm and traditional K-means algorithm for image segmentation. MSSA is a newly proposed K-means based algorithm, and other algorithms have been successfully applied to image segmentation problems in recent years. Because the K-means clustering algorithm has a strong dependence on K values, improper selection of K values will have a great impact on the results, and K-means clustering algorithm has a strong dependence on K values. Set the value of *k* to 3 to avoid interference from unrelated factors. The general parameters of the algorithm are population size of 30 and the maximum number of iterations of 100. Each algorithm divides the image as shown in Figure 5 and Figure 6. The first line in Figure 5 and Figure 6 represents the original image, and each subsequent line represents the segmentation effect of each algorithm.

It is impossible to see the difference between each algorithm in image segmentation by human eyes. Therefore, three commonly used image segmentation metrics, PSNR, SSIM, and FSIM, are selected to measure the quality of each algorithm.

Peak Signal-to-Noise Ratio (PSNR) is mainly used to measure the difference between the segmented image and the original image. The formula is as follows [57]:

(13) $$\begin{array}{c} \text{PSNR}=20.{\text{log}}_{10}\left(\frac{255}{\text{RMSE}}\right),\\ \text{RMSE}=\sqrt{\frac{\sum_{i=1}^{M}\sum_{j=1}^{Q}{\left(I\left(i,j\right)-Seg\left(i,j\right)\right)}^{2}}{M\times Q}}. \end{array}$$

In formula (12) and (13), RMSE represents the root mean square error of the pixels; *M*×*Q* represents the size of the image; *I*(*i*, *j*) represents the pixel gray value of the original image; Seg(*i*, *j*) represents the pixel gray value of the segmented image. The larger the PSNR value, the better the segmented image quality. Generally speaking, PSNR higher than 40 dB indicates excellent image quality (indicating that it is very close to the original image). At 30–40db, it usually indicates that the image quality is good (indicating that the distortion is perceptible but acceptable).

Structural Similarity (SSIM) is used to measure the similarity between the original image and the segmented image. The larger the SSIM, the better the segmented result. SSIM is defined as follows [58]:

(14) $$\begin{array}{c} \text{SSIM}=\frac{\left(2\mu_{I}\mu_{\text{seg}}+c_{1}\right)\left(2\sigma_{I,\text{seg}}+c_{2}\right)}{\left(\mu_{I}^{2}+\mu_{\text{seg}}^{2}+c_{1}\right)\left(\sigma_{I}^{2}+\sigma_{\text{seg}}^{2}+c_{2}\right)}. \end{array}$$

In formula (14), *μ*_*I*_ and *μ*_seg_ represent the average value of the original image and the segmented image; *σ*_*I*_ and *σ*_*seg*_ represent the standard deviation of the original image and the segmented image, respectively.; *σ*_*I*,seg_ represents the covariance between the original image and the segmented image; *c*_1_,  *c*_2_ are constantly used to ensure stability. SSIM value range [0,1]. The larger the value, the smaller the image distortion.

Feature similarity index mersure (FSIM) is a measure of the characteristic similarity between the original image and the quality of the segmentation, used to evaluate local structure and provide contrast information. The value range of FSIM is [0,1], and the closer the value is to 1, the better the segmentation effect. FSIM is defined as follows [59]:

(15) $$\begin{array}{c} \text{FSIM}=\frac{\sum_{l\in \Omega }S_{L}\left(X\right)PC_{m}\left(X\right)}{\sum_{l\in \Omega }PC_{m}\left(X\right)},\\ SL\left(X\right)=S_{PC}\left(X\right)S_{G}\left(X\right),\\ S_{PC}\left(X\right)=\frac{2PC_{1}\left(X\right)PC_{2}\left(X\right)+T_{1}}{PC_{1}^{2}\left(X\right)PC_{2}^{2}\left(X\right)+T_{1}},\\ PC\left(X\right)=\frac{E\left(X\right)}{\left(\varepsilon +\sum_{m}A_{n}\left(X\right)\right)}.\\ G=\sqrt{G_{x}^{2}+G_{y}^{2},}\\ S_{G}\left(X\right)=\frac{2G_{1}\left(X\right)G_{2}\left(X\right)+T_{2}}{G_{1}^{2}\left(X\right)G_{2}^{2}\left(X\right)+T_{2}}, \end{array}$$

In the above formula, Ω  is all the pixel regions of the original image; *S*_*L*_(*X*) is the similarity score; *PC*_*m*_(*X*) is the phase consistency measure; *T*_*1*_ and *T*_*2*_ are constants; *G* is the gradient descent; *E(x)* is the response vector size at position *X* and the scale is *n*; *ε* is a very small value; *An(X)* is the local size at scale *n*.

Run each algorithm 10 times, and the average and average running time of the partitioned metrics are shown in Table 8.

Simply from the naked eye, the image after IMRFO segmentation in Figures 5 and Figure 6 is clearer. Some algorithms have a rough segmentation effect and have appeared a blurry phenomenon. From Table 7, it can be seen that the segmentation index of IMRFO has a greater advantage, especially in test01 and test03-08, where more than two indexes are optimal. For example, the FSIM index in test07 reaches 0.97, SSIM in test08 reaches 0.87, which has a significant advantage over other algorithms. When the performance indicator is not optimal, IMRFO is still close to the optimal value. For example, in test01, the SSIM index of WOA is 0.7488, while that of IMRFO is 0.7479, which is close to the optimal value. In test06, the PSNR of ABC was 43.3715, and that of IMRFO was 43.1626. Therefore, both subjective visual effect and measurement result of IMRFO is better than other algorithms, which can prove a good segmentation effect. It also indirectly proves the good search performance of IMRFO, solves the problem that MRFO is easy to fall into local optimal solution and K-means has the disadvantage of being sensitive to the initial clustering center, which results in an excellent initial clustering center and further improves the image segmentation quality. On the other hand, the running time of K-means segmentation is the least, but the quality is the worst. The operation of other algorithms is large and the effect is obvious. The IMRFO does have a time disadvantage, to be expected, as it takes more time to accurately scan the solution in space.

## 7. Summary of Results

MRFO relies on group behavior to find food, so it lacks flexibility and is prone to fall into local optimum. In the existing work, most scholars can not solve such problems well. In order to improve the searching ability of MRFO, an improved algorithm for bats is presented, which uses Lévy flight, random walk learning, and learning factors.

The current experimental work is summarized as follows:

1. Comparing IMRFO with some basic algorithms on 12 standard test functions shows that the algorithm has certain advantages.
2. Two statistical tests are used to verify the universality of IMRFO and show a good search ability.
3. The convergence of each algorithm in each function is given, and the result shows that IMRFO has a good convergence rate.
4. To further verify the performance of the algorithm, IMRFO is compared with the recently proposed variants of the algorithm, and the results show that IMRFO has an obvious advantage in most functions.
5. In order to verify the validity and value of the three combinations of strategies, ablation experiments were carried out. The results show that IMRFO is better than other combinations of strategies, highlighting the practical value of IMRFO.
6. Eight underwater images were used to verify the effect of IMRFO optimized K-means image segmentation. The results show that the IMRFO optimized image segmentation quality is good and has a rational segmentation index in multiple images.

In summary, several experiments have demonstrated that IMRFO is a challenging new variant of the algorithm. IMRFO has shown good results in several test functions and image segmentation, but the optimization results in some functions and images need to be improved. More work is waiting to improve its optimization capability.

## 8. Conclusion and Future Works

In order to improve the shortcomings of K-means image segmentation and its vulnerability to local optimization, this paper presents a K-means image segmentation method based on IMRFO. IMRFO uses Lévy flight to improve the individual searchability, proposes random walk learning to prevent the premature phenomenon of the algorithm, and finally uses learning factor to improve the convergence accuracy of the algorithm so as to improve the search of the algorithm. The validity and feasibility of IMRFO are verified by 12 test functions, and through 8 underwater image data sets, it can be seen that IMRFO has a good segmentation effect and is superior to other algorithms proposed in recent years under several indicators.

Although IMRFO has good segmentation advantages in eight images, it does not achieve the best three criteria for all images. From the experimental point of view, IMRFO is only the best in test 05, while the other test pictures are basically the two best. On the other hand, the running time of each algorithm is too large, and the accuracy is at the expense of time. In the future, we will improve the image quality from the following three aspects.

1. Comprehensively improve the three performance indicators, making the three indicators the best
2. Balance the time and the search ability of the algorithm to get the best performance in an effective time
3. It can be used in agricultural, aerospace, medical, and other scenarios so that the algorithm can play a suitable role in different environments

## Figures and Tables

**Figure 1:** Lévy flight diagram.

**Figure 2:** Distribution of algorithm individuals (a) original algorithm (b) algorithm with GWL.

**Figure 3:** K-Means image segmentation based on IMRFO.

**Figure 4:** Average convergence of each algorithm.

**Figure 5:** Segmentation effect of test 01–4.

**Figure 6:** Segmentation effect of test 05–8.

**Algorithm 1:** The framework of the IMRFO.

**Table 1:** Test function information table.

F	Dim	Interval	Min
*F*_1_(*x*)=∑_*i*=1_^*n*^*x*_*i*_^2^	30/100	[-100,100]	0
*F*_2_(*x*)=∑_*i*=1_^*n*^|*x*_*i*_|+∏_*i*=1_^*n*^*x*_*i*_	30/100	[-10,10]	0
$F_{3}\left(x\right)=\overset{n}{\underset{i=1}{\sum }}{\left(\sum_{j=1}^{i}x_{j}\right)}^{2}$	30/100	[-100,100]	0
*F*_4_(*x*)=max_*i*_{|*x*_*i*_|, 1 ≤ *i* ≤ *n*}	30/100	[-100,100]	0
*F*_5_(*x*)=∑_*i*=1_^*n*−1^[100(*x*_*i*+1_ − *x*_*i*_^2^)^2^+(*x*_*i*_ − 1)^2^]	30/100	[-30,30]	0
*F*_6_(*x*)=∑_*i*=1_^*n*^*ix*_*i*_^4^+random[0,1)	30/100	[-1.28,1.28]	0
$F_{7}\left(x\right)=\sum_{i=1}^{n}-x_{i}\sin\left(\sqrt{\left|x_{i}\right|}\right)$	30/100	[-500,500]	-418.9829n
*F*_8_(*x*)=∑_*i*=1_^*n*^[*x*_*i*_^2^ − 10cos(2*πx*_*i*_)+10]	30/100	[-5.12,5.12]	0
$F_{9}\left(x\right)=-20\exp\left(-0.2\sqrt{\frac{1}{n}\sum_{i=1}^{n}x_{i}^{2}}\right)-\exp\left(\frac{1}{n}\sum_{i=1}^{n}\cos\left(2\pi x_{i}\right)\right)+20+e$	30/100	[-32,32]	0
$F_{10}\left(x\right)=\frac{1}{4000}\sum_{i=1}^{n}x_{i}^{2}-\prod_{i=1}^{n}\cos\left(\frac{x_{i}}{\sqrt{i}}\right)+1$	30/100	[-600,600]	0
*F*_11_(*x*)=(*π*/*n*){10sin(*πy*_1_)+∑_*i*=1_^*n*−1^(*y*_*i*_ − 1)^2^[1+10sin^2^(*πy*_*i*+1_)]+(*y*_*n*_ − 1)^2^}+∑_*i*=1_^*n*^*u*(*x*_*i*_, 10, 100,4)	30/100	[−50,50]	0
*y*_*i*_=1+(*x*_*i*_+1/4)			
$u\left(x_{i},a,k,m\right)=\left\{\begin{array}{cc} k{\left(x_{i}-a\right)}^{m}, & x_{i}>a,\\ 0, & -a<x_{i}<a,\\ k{\left(-x_{i}-a\right)}^{m} & x_{i}<-a. \end{array}\right.$			
*F*_12_(*x*)=(0.002+∑_*i*=1_^25^(1/*i*+(*x*_1_ − *a*_1*i*_)^6^+(*x*_2_ − *a*_2*i*_)^6^))^−1^where$a=\left(\begin{array}{cccccccccc} -32 & -16 & 0 & 16 & 32 & -32 & \ldots & 0 & 16 & 32\\ -32 & -32 & -32 & -32 & -32 & -16 & \ldots & 32 & 32 & 32 \end{array}\right)$	2	[-65.536.65.536]	0.998

**Table 2:** Performance comparison table of each algorithm

*F*	Algorithm	Best	Mean	Std
*F*_1_(*x*)	IMRFO	0	0	**0**
	MRFO	0	0	0
	HBA	9.3799*E* − 166	1.1587*E* − 160	4.2983*E* − 160
	WOA	3.1181*E* − 104	1.0841*E* − 95	4.5034*E* − 95
	TLBO	4.0530*E* − 86	2.9876*E* − 85	2.1878*E* − 85
	FPA	3.4196*E* + 04	5.6323*E* + 04	9.3090*E* + 03
	GWO	2.97266*E* − 42	9.97975*E* − 41	2.31134*E* − 40
	PSO	1.35628*E* − 12	7.30343*E* − 11	1.53846*E* − 10

*F*_2_(*x*)	IMRFO	**0**	**4.8161*E* − 277**	**0**
	MRFO	4.2592*E* − 237	1.5644*E* − 229	0
	HBA	1.0045*E* − 87	3.0642*E* − 85	8.9871*E* − 85
	WOA	5.1550*E* − 63	8.1673*E* − 58	2.9729*E* − 57
	TLBO	3.0778*E* − 43	1.2493*E* − 42	7.1358*E* − 43
	FPA	4.4336*E* + 07	7.9783*E* + 10	1.3371*E* + 11
	GWO	1.00188*E* − 24	5.16621*E* − 24	3.79647*E* − 24
	PSO	1.9394*E* − 06	1.2453*E* − 04	3.7943*E* − 04

*F*_3_(*X*)	IMRFO	**0**	**0**	**0**
	MRFO	0	4.2858*E* − 192	0
	HBA	7.5465*E* − 129	1.8442*E* − 117	6.9103*E* − 117
	WOA	4.7217*E* + 03	1.4248*E* + 04	6.9878*E* + 03
	TLBO	6.0458*E* − 17	1.7598*E* − 15	1.8686*E* − 15
	FPA	6.4669*E* + 04	9.4629*E* + 04	1.9121*E* + 04
	GWO	1.2723*E* − 15	1.6522*E* − 11	5.6380*E* − 11
	PSO	2.4597	6.8764	4.6664

*F*_4_(*X*)	IMRFO	**0**	**3.6613*E* − 283**	**0**
	MRFO	1.8994*E* − 233	1.2937*E* − 223	0
	HBA	6.4810*E* − 72	3.6559*E* − 68	8.7750*E* − 68
	WOA	1.3789*E* − 07	2.9967*E* + 01	3.0998*E* + 01
	TLBO	7.54383*E* − 35	2.2303*E* − 34	1.1471*E* − 34
	FPA	7.5982*E* + 01	8.3319*E* + 01	3.0315*E* + 00
	GWO	1.0249*E* − 11	1.3528*E* − 10	1.3630*E* − 10
	PSO	1.0009*E* + 01	1.0221*E* + 02	5.1654*E* + 01

*F*_5_(*X*)	IMRFO	1.8761*E* + 01	1.9089*E* + 01	4.2393*E* − 01
	MRFO	1.9091*E* + 01	2.0074*E* + 01	3.9236*E* − 01
	HBA	1.9310*E* + 01	2.1199*E* + 01	7.6666*E* − 01
	WOA	2.6313*E* + 01	2.6797*E* + 01	2.0942*E* − 01
	TLBO	1.6702*E* + 01	1.8846*E* + 01	1.0315
	FPA	1.0583*E* + 08	1.7478*E* + 08	3.8136*E* + 07
	GWO	4.5186*E* + 01	4.6672*E* + 01	7.8488*E* − 01
	PSO	89.4507	234.8606	104.6002

*F*_6_(*X*)	IMRFO	**1.4166*E* − 06**	**2.9500*E* − 05**	**2.0356*E* − 05**
	MRFO	3.1973*E* − 06	3.8448*E* − 05	4.0550*E* − 05
	HBA	1.6931*E* − 05	1.1151*E* − 04	8.9566*E* − 05
	WOA	3.9351*E* − 05	9.5517*E* − 04	9.4421*E* − 04
	TLBO	4.4041*E* − 04	7.9732*E* − 04	2.1545*E* − 04
	FPA	5.1790*E* + 01	9.3728*E* + 01	1.9183*E* + 01
	GWO	1.8171*E* − 04	5.6482*E* − 04	3.1680*E* − 04
	PSO	7.1930*E* − 03	1.8163*E* − 02	7.2361*E* − 03

*F*_7_(*X*)	IMRFO	−1.0536*E* + 04	−1.0050*E* + 04	4.2525*E* + 02
	MRFO	−9.6874*E* + 03	−9.0741*E* + 03	4.3594*E* + 02
	HBA	−1.0990*E* + 04	−9.4427*E* + 03	9.4018*E* + 02
	WOA	−12569.4699	−11724.03485	1302.326078
	TLBO	−9.2643*E* + 03	−7.3757*E* + 03	1.1529*E* + 03
	FPA	−4.0064*E* + 03	−2.9596*E* + 03	3.8588*E* + 02
	GWO	−8.2622*E* + 03	−6.3621*E* + 03	7.0903*E* + 02
	PSO	−8.3241*E* + 03	−6.8450*E* + 03	7.5268*E* + 02

*F*_8_(*X*)	IMRFO	**0**	**0**	**0**
	MRFO	0	0	0
	HBA	0	0	0
	WOA	0	1.8948*E* − 15	1.0378*E* − 14
	TLBO	0	6.3284	4.7427
	FPA	3.3516*E* + 02	3.9820*E* + 02	2.9755*E* + 01
	GWO	0	4.7528*E* − 01	1.4588
	PSO	0	2.0630	1.3861

*F*_9_(*X*)	IMRFO	**8.8818*E* − 16**	**8.8818*E* − 16**	**0**
	MRFO	8.8818*E* − 16	8.8818*E* − 16	0
	HBA	8.8818*E* − 16	8.8818*E* − 16	0
	WOA	8.8818*E* − 16	4.0856*E* − 15	2.6960*E* − 15
	TLBO	4.4409*E* − 15	6.3357*E* − 15	0
	FPA	1.9290*E* + 01	2.0337*E* + 01	2.7610*E* − 01
	GWO	1.8652*E* − 14	2.7652*E* − 14	3.8165*E* − 15
	PSO	1.7249*E* − 06	1.9663*E* − 01	4.5356*E* − 01

*F*_10_(*X*)	IMRFO	**0**	**0**	**0**
	MRFO	0	0	0
	HBA	0	0	0
	WOA	0	1.9723*E* − 03	3.3266*E* − 03
	TLBO	0	0	0
	FPA	2.7736*E* − 01	1.2829*E* + 00	6.1301*E* − 01
	GWO	0	2.4654*E* − 03	3.5462*E* − 03
	PSO	0	1.9723*E* − 03	3.3266*E* − 03

*F*_11_(*X*)	IMRFO	**7.3400*E* − 20**	**1.2392*E* − 18**	**1.2894*E* − 18**
	MRFO	4.04531*E* − 06	1.53518*E* − 05	8.77191*E* − 06
	HBA	3.8903*E* − 10	6.7898*E* − 09	1.1908*E* − 08
	WOA	2.7893*E* − 03	4.9054*E* − 03	1.5734*E* − 03
	TLBO	5.7527*E* − 05	2.2424*E* − 03	5.7778*E* − 03
	FPA	5.1790*E* + 07	3.7356*E* + 08	1.3609*E* + 08
	GWO	1.4152*E* − 06	1.4681*E* − 02	9.2775*E* − 03
	PSO	6.4838*E* − 14	8.6436*E* − 02	2.5276*E* − 01

*F*_12_(*X*)	IMRFO	**9.9800*E* − 01**	**9.9800*E* − 01**	**0**
	MRFO	9.9800*E* − 01	9.9800*E* − 01	0
	HBA	9.9800*E* − 01	9.9800*E* − 01	0
	WOA	9.9800*E* − 01	1.2626	6.8599*E* − 01
	TLBO	9.9800*E* − 01	9.9800*E* − 01	0
	FPA	1.9995	1.0262*E* + 01	7.6364
	GWO	9.9800*E* − 01	1.7255*E* + 00	9.7247*E* − 01
	PSO	9.9800*E* − 01	1.1305*E* + 00	3.4368*E* − 01

The optimal value is shown in bold.

**Table 3:** Table of results for each algorithm (100 DIMENSIONS).

F	Algorithm	Best	Mean	Std
F_1_(x)	IMRFO	**0**	**0**	**0**
	MRFO	0	0	0
	HBA	8.9040E-147	4.6592E-141	1.2550E-140
	WOA	1.0469E-102	7.2231E-93	2.5499E-92
	TLBO	1.6114E-75	1.6114E-75	1.1585E-75
	FPA	1.3848 E+05	2.2811 E+05	4.4746 E+04
	GWO	5.0821E-18	2.6308E-17	2.1090E-17
	PSO	1.0669	1.2459 E+01	3.0029 E+01

F_2_(x)	IMRFO	**2.0908E-305**	**4.0935E-281**	**0**
	MRFO	8.2591E-234	8.7997E-228	0
	HBA	3.2693E-78	1.4848E-75	2.1169E-75
	WOA	3.97136E-62	8.1673E-58	4.04975E-55
	TLBO	1.58996E-38	1.11006E-55	1.64669E-38
	FPA	2.5777 E+27	4.8007 E+45	1.3669 E+46
	GWO	1.1188E-23	1.0071E-22	8.1329E-23
	PSO	1.6825E-06	4.0865E-05	1.3518E-04
F_3_(X)	IMRFO	**0**	**0**	0
	MRFO	0	4.2858E-192	0
	HBA	5.8574E-106	6.5344E-94	3.2931E-93
	WOA	4.5880 E+05	6.7389 E+05	1.1901E+05
	TLBO	5.7047E-06	1.4581E-04	1.5072E-04
	FPA	5.9828 E+05	9.8255 E+05	2.2421 E+05
	GWO	4.3996E-01	1.1814 E+01	1.3585 E+01
	PSO	4.1855 E+03	6.8320 E+03	7.6320 E+03

F_4_(X)	IMRFO	**2.0908E-305**	**4.0728E-281**	**0**
	MRFO	1.0891E-224	6.0212E-219	0
	HBA	4.1580E-49	6.4459E-47	1.2824E-46
	WOA	9.9712E-04	7.4068 E+01	2.9309 E+01
	TLBO	2.64171E-30	4.63468E-30	1.35657E-30
	FPA	8.7604 E+01	9.3681 E+01	2.0880
	GWO	2.0983E-03	5.2094E-02	8.6554E-02
	PSO	7.3783	9.5754	1.2668

F_5_(X)	IMRFO	**9.0554 E+01**	9.1195 E+01	7.3432E-01
	MRFO	9.0823 E+01	9.2361 E+01	6.6140E-01
	HBA	9.1619 E+01	9.4762 E+01	1.8652 E+00
	WOA	9.6679 E+01	9.7258 E+01	3.0684E-01
	TLBO	9.1198 E+01	9.3064 E+01	9.5488E-01
	FPA	4.0625 E+08	9.3161 E+08	2.3879 E+08
	GWO	9.5679 E+01	9.6973 E+01	9.2081E-01
	PSO	6.5109 E+02	3.2217 E+03	6.7489 E+03

F_6_(X)	IMRFO	**1.4328E-06**	**6.6842E-05**	4.9030E-05
	MRFO	2.0781E-06	4.9605E-05	4.3316E-05
	HBA	2.3868E-05	1.4383E-04	1.2534E-04
	WOA	8.5089E-06	1.3208E-03	1.3226E-03
	TLBO	5.1751E-04	1.1234E-03	3.2954E-04
	FPA	6.1163 E+02	1.4259 E+03	3.5171 E+02
	GWO	9.4824E-04	2.6521E-03	1.1372E-03
	PSO	4.9985E-01	1.1220 E+00	3.6320E-01

F_7_(X)	IMRFO	-2.92 E+04	-2.57 E+04	1.67 E+03
	MRFO	-2.7791 E+04	-2.5142 E+04	1.1769 E+03
	HBA	-3.2530 E+04	-2.6092 E+04	3.5550 E+03
	WOA	-4.1898 E+04	-3.9015 E+04	3.7697 E+03
	TLBO	-2.7940 E+04	-1.6598 E+04	5.1640 E+03
	FPA	-6.5597 E+03	-5.3592 E+03	6.0949 E+02
	GWO	-2.2404 E+04	-1.6607 E+04	2.4372 E+03
	PSO	-2.3436 E+04	-2.0057 E+04	2.2771 E+03

F_8_(X)	IMRFO	**0**	**0**	0
	MRFO	0	0	0
	HBA	0	0	0
	WOA	0	3.7896E-15	2.0756E-14
	TLBO	0	6.3284	4.7427
	FPA	1.3434 E+03	1.5311 E+03	8.6281 E+01
	GWO	0	1.3971	2.2329
	PSO	2.8854 E+01	4.8456 E+01	1.1153 E+01

F_9_(X)	IMRFO	**8.8818E-16**	**8.8818E-16**	**0**
	MRFO	8.8818E-16	8.8818E-16	0
	HBA	8.8818E-16	8.8818E-16	0
	WOA	8.8818E-16	4.3225E-15	2.8731E-15
	TLBO	7.9936E-15	7.9936E-15	0
	FPA	1.9841 E+01	2.0520 E+01	3.3562E-01
	GWO	2.2204E-14	3.0257E-14	3.7242E-15
	PSO	1.3320E-06	1.4424E-01	4.4254E-01

F_10_(X)	IMRFO	**0**	**0**	0
	MRFO	0	0	0
	HBA	0	0	0
	WOA	0	0	0
	TLBO	0	0	0
	FPA	1.3815 E+03	2.0376 E+03	3.4470 E+02
	GWO	0	1.8958E-03	3.1773E-03
	PSO	0	1.3192E-03	2.8042E-03

F_11_(X)	IMRFO	**2.8193E-06**	**6.4940E-06**	**3.2213E-06**
	MRFO	4.6460E-06	1.09637E-05	6.3630E-06
	HBA	1.9642E-02	3.5856E-02	1.0354E-02
	WOA	1.8029E-03	7.0382E-03	9.1277E-03
	TLBO	7.3698E-05	2.3727E-03	5.8937E-03
	FPA	7.4824 E+08	2.1393 E+09	7.0466 E+08
	GWO	2.1287E-06	1.5932E-02	9.1126E-03
	PSO	2.3297E-13	8.2984E-02	1.7745E-01

F_12_(X)	IMRFO	**9.9800E-01**	**9.9800E-01**	**0**
	MRFO	9.9800E-01	9.9800E-01	0
	HBA	9.9800E-01	9.9800E-01	0
	WOA	9.9800E-01	1.2626	6.8599E-01
	TLBO	9.9800E-01	9.9800E-01	0
	FPA	1.9995	1.0262 E+01	7.6364
	GWO	9.9800E-01	1.7255 E+00	9.7247E-01
	PSO	9.9800E-01	1.1305 E+00	3.4368E-01

Bold font is to clearly see the advantages of the algorithm. The best indicators of IMRFO have been bold in this paper.

**Table 4:** Wilcoxon rank-sum test *p*-value.

F	MRFO	FPA	GWO	HBA	PSO	TLBO	WOA
F1	N/A	1.21E-12	1.21E-12	1.21E-12	1.21E-12	1.21E-12	1.21E-12
F2	3.02E-11	3.02E-11	3.02E-11	3.02E-11	3.02E-11	3.02E-11	3.02E-11
F3	N/A	1.21E-12	1.21E-12	1.21E-12	1.21E-12	1.21E-12	1.21E-12
F4	3.02E-11	3.02E-11	3.02E-11	3.02E-11	3.02E-11	3.02E-11	3.02E-11
F5	1.46E-09	1.79E-11	1.79E-11	4.94E-11	3.53E-10	N/A	1.79E-11
F6	N/A	2.91E-11	2.91E-11	5.07E-07	2.91E-11	2.91E-11	2.29E-10
F7	7.61E-09	1.44E-11	1.44E-11	3.31E-03	1.44E-11	1.97E-11	7.40E-07
F8	N/A	1.21E-12	8.15E-02	N/A	4.24E-12	1.66E-11	3.34E-01
F9	N/A	1.21E-12	6.59E-13	N/A	1.21E-12	4.63E-13	1.02E-07
F10	N/A	1.21E-12	6.62E-04	N/A	1.35E-03	N/A	2.79E-03
F11	3.02E-11	3.02E-11	3.02E-11	3.02E-11	3.02E-11	3.02E-11	3.02E-11
F12	5.46E-03	1.14E-11	1.14E-11	4.95E-10	6.79E-02	2.50E-05	1.14E-11

**Table 5:** Friedman test ranking table.

Algorithms	IMRFO	MRFO	HBA	WOA	TLBO	FPA	GWO	PSO
Rank	2.0208	2.2708	2.8333	5.0000	4.4583	7.5417	5.4167	6.4583

**Table 6:** Comparison with variants of the algorithm

*F*	Algorithm	Best	Mean	Std
*F*_1_(*x*)	IMRFO	**0**	**0**	**0**
	FACL	2.6020*E* + 02	2.6020*E* + 02	4.5704*E* − 13
	MSSCS	2.6586*E* − 16	1.2320*E* − 14	2.2109*E* − 14
	SACS	5.8993*E* − 17	2.1975*E* − 15	2.2919*E* − 15
	CSsin	8.1279*E* − 17	1.8682*E* − 15	2.2000*E* − 15

*F*_2_(*x*)	IMRFO	**0**	**4.8161*E* − 277**	**0**
	FACL	1.3615*E* + 01	1.3615*E* + 01	1.7853*E* − 15
	MSSCS	2.4907*E* − 09	1.0918*E* − 08	9.6029*E* − 09
	SACS	8.1604*E* − 10	3.6463*E* − 09	2.3128*E* − 09
	CSsin	8.7299*E* − 10	3.3430*E* − 09	1.7651*E* − 09

*F*_3_(*X*)	IMRFO	**0**	**0**	**0**
	FACL	2.3244*E* + 03	2.3244*E* + 03	2.7422*E* − 12
	MSSCS	2.1933*E* − 02	6.6588*E* − 01	1.2328*E* + 00
	SACS	2.0617*E* − 13	4.2875*E* − 10	7.7897*E* − 10
	CSsin	3.4984*E* − 13	3.5258*E* − 09	1.8741*E* − 08

*F*_4_(*X*)	IMRFO	**0**	**3.6613*E* − 283**	**0**
	FACL	1.5622*E* + 01	1.5622*E* + 01	1.4282*E* − 14
	MSSCS	9.5018*E* − 05	2.8057*E* − 03	7.0418*E* − 03
	SACS	2.5496*E* − 15	2.8163*E* − 12	8.9570*E* − 12
	CSsin	1.1423*E* − 15	1.3641*E* − 12	4.9902*E* − 12

*F*_5_(*X*)	IMRFO	1.8761*E* + 01	1.9089*E* + 01	4.2393*E* − 01
	FACL	6.2978*E* + 04	6.2978*E* + 04	7.3126*E* − 11
	MSSCS	2.1186*E* + 01	2.6991*E* + 01	1.5287*E* + 01
	SACS	9.5265*E* − 03	1.6347*E* + 01	1.0434*E* + 01
	CSsin	3.1439*E* + 00	1.4000*E* + 01	4.5249*E* + 00

*F*_6_(*X*)	IMRFO	**1.4166*E* − 06**	**2.9500*E* − 05**	**2.0356*E* − 05**
	FACL	4.9638*E* − 01	2.6540*E* + 00	3.6836*E* + 00
	MSSCS	1.0931*E* − 03	3.7296*E* − 03	1.7917*E* − 03
	SACS	2.7015*E* − 04	1.2413*E* − 03	6.5230*E* − 04
	CSsin	2.5773*E* − 04	1.2047*E* − 03	6.2553*E* − 04

*F*_7_(*X*)	IMRFO	−1.0536*E* + 04	−1.0050*E* + 04	4.2525*E* + 02
	FACL	−3.2588*E* + 03	−3.2588*E* + 03	3.6563*E* − 12
	MSSCS	−1.2409*E* + 04	−1.2023*E* + 04	1.7642*E* + 02
	SACS	−1.2337*E* + 04	−1.2040*E* + 04	1.6571*E* + 02
	CSsin	−1.2197*E* + 04	−1.1773*E* + 04	2.2010*E* + 02

*F*_8_(*X*)	IMRFO	**0**	**0**	**0**
	FACL	1.3469*E* + 02	1.3469*E* + 02	1.9995*E* − 13
	MSSCS	1.3682*E* + 02	1.3682*E* + 02	2.2852*E* − 13
	SACS	1.3558*E* + 01	1.9318*E* + 01	3.2639*E* + 00
	CSsin	1.3082*E* + 01	1.7173*E* + 01	2.4068*E* + 00

*F*_9_(*X*)	IMRFO	**8.8818*E* − 16**	**8.8818*E* − 16**	**0**
	FACL	9.5803*E* + 00	9.5803*E* + 00	1.4282*E* − 14
	MSSCS	7.8366*E* − 09	3.3808*E* − 08	2.3225*E* − 08
	SACS	6.6614*E* − 09	3.5846*E* − 08	2.6071*E* − 08
	CSsin	9.4992*E* − 09	4.9013*E* − 08	3.5110*E* − 08

*F*_10_(*X*)	IMRFO	**0**	**0**	**0**
	FACL	1.6979*E* + 01	1.6979*E* + 01	2.4994*E* − 14
	MSSCS	6.6613*E* − 16	8.2473*E* − 04	4.4988*E* − 03
	SACS	1.6653*E* − 15	3.2272*E* − 03	9.0416*E* − 03
	CSsin	6.6613*E* − 16	1.8055*E* − 03	8.5946*E* − 03

*F*_11_(*X*)	IMRFO	**7.3400*E* − 20**	**1.2392*E* − 18**	**1.2894*E* − 18**
	FACL	8.7100*E* + 00	8.7100*E* + 00	1.4282*E* − 14
	MSSCS	1.5139*E* − 07	5.4848*E* − 07	3.2760*E* − 07
	SACS	2.2637*E* − 07	4.8725*E* − 07	3.3696*E* − 07
	CSsin	1.7143*E* − 07	5.0219*E* − 07	3.9414*E* − 07

*F*_12_(*X*)	IMRFO	**9.9800*E* − 01**	**9.9800*E* − 01**	**0**
	FACL	1.9920*E* + 00	1.9920*E* + 00	4.4633*E* − 15
	MSSCS	—	—	—
	SACS	9.9800*E* − 01	9.9800*E* − 01	0
	CSsin	9.9800*E* − 01	9.9800*E* − 01	0

The optimal value is shown in bold.

**Table 7:** Test table for each combination algorithm.

F	Algorithm	Best	Mean	Std
F_1_(x)	IMRFO	**0**	**0**	**0**
	MRFO-I	0	0	0
	MRFO-II	0	0	0
	MRFO-III	0	0	0
	MRFO-IV	0	0	0
	MRFO-V	0	0	0
	MRFO-VI	0	0	0

F_2_(x)	IMRFO	**0**	**4.8161E-277**	**0**
	MRFO-I	2.2366E-239	2.3660E-230	0
	MRFO-II	1.4788E-239	3.6180E-231	0
	MRFO-III	6.7519E-240	2.1114E-231	0
	MRFO-IV	4.9710E-237	1.7202E-229	0
	MRFO-V	3.4101E-236	1.0691E-229	0
	MRFO-VI	6.6058E-239	8.1070E-230	0

F_3_(X)	IMRFO	**0**	**0**	**0**
	MRFO-I	0	0	0
	MRFO-II	0	0	0
	MRFO-III	0	0	0
	MRFO-IV	0	0	0
	MRFO-V	0	0	0
	MRFO-VI	0	0	0

F_4_(X)	IMRFO	**0**	**3.6613E-283**	**0**
	MRFO-I	7.1957E-231	9.1743E-224	0
	MRFO-II	5.5959E-232	2.5385E-224	0
	MRFO-III	2.2845E-232	2.3915E-224	0
	MRFO-IV	1.7079E-231	6.1960E-224	0
	MRFO-V	3.1285E-233	3.7719E-225	2.0880
	MRFO-VI	3.3266E-233	2.8006E-224	8.6554E-02

F_5_(X)	IMRFO	**1.8761 E+01**	**1.9089 E+01**	4.2393E-01
	MRFO-I	1.9160 E+01	2.0228 E+01	4.7486E-01
	MRFO-II	1.9205 E+01	1.9904 E+01	4.1531E-01
	MRFO-III	1.9050 E+01	2.0040 E+01	4.5484E-01
	MRFO-IV	1.9054 E+01	1.9923 E+01	4.8479E-01
	MRFO-V	1.8959 E+01	2.0027 E+01	5.1658E-01
	MRFO-VI	1.8883 E+01	1.9994 E+01	6.7667E-01

F_6_(X)	IMRFO	**1.4166E-06**	**2.9500E-05**	**2.0356E-05**
	MRFO-I	3.3254E-06	4.0901E-05	2.9878E-05
	MRFO-II	1.7086E-06	4.2369E-05	3.8592E-05
	MRFO-III	2.9884E-06	4.3133E-05	4.4862E-05
	MRFO-IV	5.3342E-06	5.1792E-05	5.3359E-05
	MRFO-V	8.3930E-06	6.0626E-05	4.2128E-05
	MRFO-VI	4.8785E-06	5.3014E-05	4.7227E-05

F_7_(X)	IMRFO	**-1.0536 E+04**	**-1.0050 E+04**	**4.2525 E+02**
	MRFO-I	-9.7467 E+03	-8.7240 E+03	6.4405 E+02
	MRFO-II	-9.9243 E+03	-8.7951 E+03	6.3557 E+02
	MRFO-III	-9.8848 E+03	-8.8964 E+03	5.5148 E+02
	MRFO-IV	-1.0102 E+04	-8.7470 E+03	6.3365 E+02
	MRFO-V	-1.0359 E+04	-8.9240 E+03	7.0323 E+02
	MRFO-VI	-1.0082 E+04	-9.0438 E+03	5.6962 E+02

F_8_(X)	IMRFO	**0**	**0**	**0**
	MRFO-I	0	0	0
	MRFO-II	0	0	0
	MRFO-III	0	0	0
	MRFO-IV	0	0	0
	MRFO-V	0	0	0
	MRFO-VI	0	0	0

F_9_(X)	IMRFO	**8.8818E-16**	**8.8818E-16**	**0**
	MRFO-I	8.8818E-16	8.8818E-16	0
	MRFO-II	8.8818E-16	8.8818E-16	0
	MRFO-III	8.8818E-16	8.8818E-16	0
	MRFO-IV	8.8818E-16	8.8818E-16	0
	MRFO-V	8.8818E-16	8.8818E-16	0
	MRFO-VI	8.8818E-16	8.8818E-16	0

F_10_(X)	IMRFO	**0**	**0**	**0**
	MRFO-I	0	0	0
	MRFO-II	0	0	0
	MRFO-III	0	0	0
	MRFO-IV	0	0	0
	MRFO-V	0	0	0
	MRFO-VI	0	0	0

F_11_(X)	IMRFO	**7.3400E-20**	1.2392E-18	1.2894E-18
	MRFO-I	1.9606E-19	1.5295E-18	1.7575E-18
	MRFO-II	1.8111E-19	1.4964E-18	1.1884E-18
	MRFO-III	1.2951E-19	2.0136E-18	2.1218E-18
	MRFO-IV	3.8758E-19	2.7853E-18	4.2987E-18
	MRFO-V	1.1870E-19	1.1469E-18	1.0703E-18
	MRFO-VI	9.2691E-20	1.8700E-18	2.1327E-18

F_12_(X)	IMRFO	**9.9800E-01**	**9.9800E-01**	**0**
	MRFO-I	9.9800E-01	9.9800E-01	0
	MRFO-II	9.9800E-01	9.9800E-01	0
	MRFO-III	9.9800E-01	9.9800E-01	0
	MRFO-IV	9.9800E-01	9.9800E-01	0
	MRFO-V	9.9800E-01	9.9800E-01	0
	MRFO-VI	9.9800E-01	9.9800E-01	0

Bold font is to clearly see the advantages of the algorithm.

**Table 8:** Segmentation effect tables for each algorithm.

Image	Index	K-means	PSO	MRFO	DPSO	MSSA	IMRFO
Test 01	PSNR	8.0602	42.9051	42.9934	42.8040	43.4789	**44.4989**
	SSIM	0.0525	0.7354	0.7412	0.7370	0.7671	0.7479
	FSIM	0.5556	0.9478	0.9476	0.9571	0.9467	**0.9579**
	Ave time	**2.5886**	39.2606	76.7789	38.4986	50.6846	76.3475

Test 02	PSNR	6.4532	44.0008	43.3155	44.0595	43.9037	43.7004
	SSIM	0.0306	0.7975	0.7788	**0.8027**	0.7877	0.7970
	FSIM	0.4934	0.9464	0.9473	0.9410	0.9508	**0.9601**
	Ave time	**5.9745**	43.9744	78.42064	38.7315	50.7706	74.5214

Test 03	PSNR	6.6314	43.1602	43.3925	43.3760	43.2782	**43.7128**
	SSIM	0.0273	0.7615	0.7770	0.7655	0.7678	**0.7894**
	FSIM	0.4249	0.9400	0.9470	0.9424	**0.9506**	0.9430
	Ave time	**2.4941**	42.6951	75.7196	38.5346	50.7550	74.7570

Test 04	PSNR	7.6085	43.0707	42.7419	43.2700	42.6999	43.1534
	SSIM	0.0461	0.7559	0.7396	0.7651	0.7380	**0.7808**
	FSIM	0.4920	0.9351	0.9435	0.9334	0.9397	**0.9466**
	Ave time	**5.8564**	41.2824	77.9430	38.4732	52.1376	75.2728

Test 05	PSNR	7.7941	43.1295	42.9913	43.2999	42.6999	**43.5453**
	SSIM	0.0187	0.7542	0.7503	0.7637	0.7380	**0.7726**
	FSIM	0.4011	0.9551	0.9566	0.9596	0.9397	**0.9634**
	Ave time	**2.2253**	37.4426	73.5829	37.6144	48.2604	73.7482

Test 06	PSNR	9.6892	42.9705	42.7052	43.539	42.8316	43.1626
	SSIM	0.0393	0.7375	0.7309	0.7385	0.7338	**0.7517**
	FSIM	0.5301	0.9501	0.9567	0.9480	0.9474	**0.9604**
	Ave time	**1.2299**	37.5475	72.6558	39.0477	48.7618	74.5432

Test 07	PSNR	7.82	42.7995	42.8791	72.8223	42.7924	**43.0107**
	SSIM	0.1071	0.7357	0.7399	0.7377	0.7414	0.7409
	FSIM	0.4460	0.9625	0.9584	0.9667	0.9558	**0.9734**
	Ave time	**2.3464**	39.1573	74.3283	38.1076	49.2879	74.5704

Test 08	PSNR	8.2165	44.1114	43.5191	44.5560	42.8239	**46.4141**
	SSIM	0.0210	0.7681	0.7417	0.7835	0.7185	**0.8710**
	FSIM	0.6614	0.8259	0.8130	0.8064	0.8444	0.8340
	Ave time	**1.2530**	38.8315	74.7158	38.2203	48.7720	75.4689

*F*	*index*	*WOA*	*ABC*	*TLBO*	*FPA*	*SSA*	*IMRFO*

Test 01	PSNR	43.1176	43.1018	42.8136	43.0370	43.4300	**44.4989**
	SSIM	**0.7488**	0.7473	0.7341	0.7407	0.7545	0.7479
	FSIM	0.9476	0.9441	0.9438	0.9441	0.9466	**0.9579**
	ave time	38.3036	39.4908	74.8217	40.1402	39.1653	76.3475

Test 02	PSNR	**44.1919**	43.5238	43.4408	42.9663	43.4401	43.7004
	SSIM	**0.8006**	0.7836	0.7852	0.7622	0.7808	0.7970
	FSIM	0.9482	0.9585	0.9557	0.9487	0.9531	**0.9601**
	ave time	38.8852	40.4172	75.3121	39.2922	42.0149	74.5214

Test 03	PSNR	43.4085	43.4408	43.0703	43.2635	43.3470	**43.7128**
	SSIM	0.7746	0.7790	0.7641	0.7731	0.7738	**0.7894**
	FSIM	0.9422	0.9453	0.9452	0.9442	0.9503	0.9430
	ave time	38.7937	42.8378	75.0803	41.8402	40.2512	74.7570

Test 04	PSNR	**43.3877**	43.2727	43.2877	42.7467	42.4343	43.1534
	SSIM	0.7600	0.7622	0.7630	0.7410	0.7256	**0.7808**
	FSIM	0.9426	0.9402	0.9403	0.9400	0.9380	**0.9466**
	ave time	39.2289	40.4403	74.4058	39.5984	39.0673	75.2728

Test 05	PSNR	42.9238	42.9262	42.9594	42.8405	42.9593	**43.5453**
	SSIM	0.7518	0.7514	0.7497	0.7480	0.7497	**0.7726**
	FSIM	0.9607	0.9605	0.9568	0.9586	0.9568	**0.9634**
	ave time	39.0783	38.9743	74.9810	38.6717	40.5572	73.7482

Test 06	PSNR	42.9003	**43.3715**	42.5365	42.5136	43.1584	43.1626
	SSIM	0.7356	0.7501	0.7107	0.7147	10.7503	**0.7517**
	FSIM	0.9396	0.9503	0.9444	0.9442	0.9511	**0.9604**
	ave time	37.5257	38.4848	76.3897	38.1784	37.8186	74.5432

Test 07	PSNR	42.8455	42.8353	42.8986	42.8399	42.8093	**43.0107**
	SSIM	0.7410	0.7386	0.7409	**0.7450**	0.7397	0.7409
	FSIM	0.9426	0.9551	0.9566	0.9367	0.9491	**0.9734**
	ave time	38.7532	39.6091	74.4956	38.6593	38.118674	74.5704

Test 08	PSNR	44.0623	45.5442	43.2560	45.3984	43.7115	**46.4141**
	SSIM	0.7663	0.8221	0.7315	0.8182	0.7545	**0.8710**
	FSIM	0.8381	0.8398	0.8196	0.8263	0.8316	0.8340
	ave time	39.3148	39.1180	76.6363	39.1871	38.8752	75.4689

The bold font here is to see the advantages and disadvantages of IMRFO. Although IMRFO has good performance, it has no advantage in time.

## Data Availability

Some data of this study are confidential, so the experimental data cannot be uploaded. These data can be obtained from the corresponding author on request.

## References

[1] Ardizzone E., Pirrone R., Gambino O. Fuzzy c-means segmentation on brain mr slices corrupted by rf-inhomogeneity.

[2] Li W., Wang G.-G., Gandomi A. H. (2021). A survey of learning-based intelligent optimization algorithms. *Archives of Computational Methods in Engineering*.

[3] Hrosik R. C., Tuba E., Dolicanin E., Jovanovic R., Tuba M. (2019). Brain image segmentation based on firefly algorithm combined with k-means clustering. *Studies in Informatics and Control*.

[4] Li H., He H., Wen Y. (2015). Dynamic particle swarm optimization and K-means clustering algorithm for image segmentation. *Optik*.

[5] Mirjalili S., Mirjalili S. M., Lewis A. (2014). Grey wolf optimizer. *Advances in Engineering Software*.

[6] Kapoor S., Zeya I., Singhal C., Nanda S. J. (2017). A grey wolf optimizer based automatic clustering algorithm for satellite image segmentation. *Procedia Computer Science*.

[7] Wang G.-G., Deb S., Cui Z. (2019). Monarch butterfly optimization. *Neural Computing & Applications*.

[8] Wang G.-G, Deb S., Coelho L. D. S. Elephant herding optimization.

[9] Wang G.-G. (2018). Moth search algorithm: a bio-inspired metaheuristic algorithm for global optimization problems. *Memetic Computing*.

[10] Heidari A. A., Mirjalili S., Faris H., Aljarah I., Mafarja M., Chen H. (2019). Harris hawks optimization: algorithm and applications. *Future Generation Computer Systems*.

[11] Kennedy J., Eberhart R. C. A discrete binary version of the particle swarm algorithm.

[12] Xia X., Gui L., Yu F. (2019). Triple archives particle swarm optimization. *IEEE Transactions on Cybernetics*.

[13] Whitley D. (1994). A genetic algorithm tutorial. *Statistics and Computing*.

[14] Liu S.-C., Chen Z.-G., Zhan Z.-H., Jeon S.-W., Kwong S., Zhang J. (2021). Many-objective job-shop scheduling: a multiple populations for multiple objectives-based genetic algorithm approach. *IEEE Transactions on Cybernetics*.

[15] Das S., Ponnuthurai N. S. (2010). Differential evolution: a survey of the state-of-the-art. *IEEE Transactions on Evolutionary Computation*.

[16] Zhan Z. H., Wang Z. J., Jin H., Zhang J. (2019). Adaptive distributed differential evolution. *IEEE Transactions on Cybernetics*.

[17] Yang X. S., Deb S. Cuckoo search via Lévy flights.

[18] Rashedi E., Nezamabadi-Pour H., Saryazdi S. (2009). GSA: a gravitational search algorithm. *Information Sciences*.

[19] Karaboga D., Basturk B. (2008). On the performance of artificial bee colony (ABC) algorithm. *Applied Soft Computing*.

[20] Zhao W., Zhang Z., Wang L. (2020). Manta ray foraging optimization: an effective bio-inspired optimizer for engineering applications. *Engineering Applications of Artificial Intelligence*.

[21] Fathy A., Rezk H., Yousri D. (2020). A robust global MPPT to mitigate partial shading of triple-junction solar cell-based system using manta ray foraging optimization algorithm. *Solar Energy*.

[22] Houssein E. H., Zaki G. N., Diab A. A. Z., Younis E. M. (2021). An efficient Manta Ray Foraging Optimization algorithm for parameter extraction of three-diode photovoltaic model. *Computers & Electrical Engineering*.

[23] Houssein E. H., Ibrahim I. E., Neggaz N., Hassaballah M., Wazery Y. M. (2021). An efficient ECG arrhythmia classification method based on Manta ray foraging optimization. *Expert Systems with Applications*.

[24] Aly M., Rezk H. (2021). A MPPT based on optimized FLC using manta ray foraging optimization algorithm for thermo‐electric generation systems. *International Journal of Energy Research*.

[25] Hemeida M. G., Ibrahim A. A., Mohamed A.-A. A., Alkhalaf S., El-Dine A. M. B. (2021). Optimal allocation of distributed generators DG based Manta Ray Foraging Optimization algorithm (MRFO). *Ain Shams Engineering Journal*.

[26] Hemeida M. G., Alkhalaf S., Mohamed A.-A. A., Ibrahim A. A., Senjyu T. (2020). Distributed generators optimization based on multi-objective functions using manta rays foraging optimization algorithm (MRFO). *Energies*.

[27] Shaheen A. M., Ginidi A. R., El-Sehiemy R. A., Ghoneim S. S. M. (2020). Economic power and heat dispatch in cogeneration energy systems using manta ray foraging optimizer. *IEEE Access*.

[28] Ben U. C., Akpan A. E., Mbonu C. C., Ebong E. D. (2021). Novel methodology for interpretation of magnetic anomalies due to two-dimensional dipping dikes using the Manta Ray Foraging Optimization. *Journal of Applied Geophysics*.

[29] Akdag O., Yeroglu C. (2021). Optimal directional overcurrent relay coordination using MRFO algorithm: a case study of adaptive protection of the distribution network of the Hatay province of Turkey. *Electric Power Systems Research*.

[30] Ghosh K. K., Guha R., Bera S. K., Kumar N., Sarkar R. (2021). S-shaped versus V-shaped transfer functions for binary Manta ray foraging optimization in feature selection problem. *Neural Computing & Applications*.

[31] A Alturki F., Mh Farh H., A Al-Shamma’a A., AlSharabi K. (2020). Techno-economic optimization of small-scale hybrid energy systems using manta ray foraging optimizer. *Electronics*.

[32] Elmaadawy K., Abd Elaziz M., Elsheikh A. H., Moawad A., Liu B., Lu S. (2021). Utilization of random vector functional link integrated with manta ray foraging optimization for effluent prediction of wastewater treatment plant. *Journal of Environmental Management*.

[33] Abd Elaziz M., Yousri D., Al-qaness M. A., AbdelAty A. M., Radwan A. G., Ewees A. A. (2021). A Grunwald–Letnikov based Manta ray foraging optimizer for global optimization and image segmentation. *Engineering Applications of Artificial Intelligence*.

[34] Hassan M. H., Houssein E. H., Mahdy M. A., Kamel S. (2021). An improved manta ray foraging optimizer for cost-effective emission dispatch problems. *Engineering Applications of Artificial Intelligence*.

[35] Xu H., Song H., Xu C., Wu X., Yousefi N. (2020). Exergy analysis and optimization of a HT-PEMFC using developed manta ray foraging optimization algorithm. *International Journal of Hydrogen Energy*.

[36] Houssein E. H., Emam M. M., Ali A. A. (2021). Improved manta ray foraging optimization for multi-level thresholding using COVID-19 CT images. *Neural Computing & Applications*.

[37] Jena B., Naik M. K., Panda R., Abraham A. (2021). Maximum 3D Tsallis entropy based multilevel thresholding of brain MR image using attacking Manta Ray foraging optimization. *Engineering Applications of Artificial Intelligence*.

[38] Micev M., Ćalasan M., Ali Z. M., Hasanien H. M., Abdel Aleem S. H. E. (2021). Optimal design of automatic voltage regulation controller using hybrid simulated annealing - manta ray foraging optimization algorithm. *Ain Shams Engineering Journal*.

[39] Ekinci S., Izci D., Hekimoğlu B. (2021). Optimal FOPID speed control of DC motor via opposition-based hybrid manta ray foraging optimization and simulated annealing algorithm. *Arabian Journal for Science and Engineering*.

[40] Haklı H. ., Uğuz H. (2014). A novel particle swarm optimization algorithm with Levy flight. *Applied Soft Computing*.

[41] Jensi R., Jiji G. W. (2016). An enhanced particle swarm optimization with levy flight for global optimization. *Applied Soft Computing*.

[42] Liu Y., Cao B. (2020). A novel ant colony optimization algorithm with Levy flight. *IEEE Access*.

[43] Li X., Engelbrecht A., Epitropakis M. G. (2013). *Benchmark functions for CEC’2013 special session and competition on niching methods for multimodal function optimization*.

[44] Molga M., Smutnicki C. (2005). Test functions for optimization needs. *Test Functions for Optimization Needs*.

[45] Hashim F. A., Houssein E. H., Hussain K., Mabrouk M. S., Al-Atabany W. (2022). Honey Badger Algorithm: new metaheuristic algorithm for solving optimization problems. *Mathematics and Computers in Simulation*.

[46] Mirjalili S., Lewis A. (2016). The whale optimization algorithm. *Advances in Engineering Software*.

[47] Rao R. V., Savsani V. J., Vakharia D. P. (2011). Teaching-learning-based optimization: a novel method for constrained mechanical design optimization problems. *Computer-Aided Design*.

[48] Yang X.-S. Flower pollination algorithm for global optimization.

[49] Demšar J. (2006). Statistical comparisons of classifiers over multiple data sets. *Journal of Machine Learning Research*.

[50] Peng H., Zeng Z., Deng C., Wu Z. (2021). Multi-strategy serial cuckoo search algorithm for global optimization. *Knowledge-Based Systems*.

[51] Peng H., Zhu W., Deng C., Wu Z. (2021). Enhancing firefly algorithm with courtship learning. *Information Sciences*.

[52] Salgotra R., Singh U., Saha S., Gandomi A. H. (2021). Self adaptive cuckoo search: analysis and experimentation. *Swarm and Evolutionary Computation*.

[53] Salgotra R., Singh U., Saha S., Gandomi A. H. Improving cuckoo search: incorporating changes for CEC 2017 and CEC 2020 benchmark problems.

[54] Islam M., Luo P., Sattar J. (2020). Simultaneous enhancement and super-resolution of underwater imagery for improved visual perception. https://www.semanticscholar.org/paper/Simultaneous-Enhancement-and-Super-Resolution-of-Islam-Luo.

[55] Xue J., Shen B. (2020). A novel swarm intelligence optimization approach: sparrow search algorithm. *Systems Science & Control Engineering*.

[56] Chen G., Dong L., Dong C., Chen X. (2021). Image segmentation based on logistic regression sparrow algorithm. *Journal of Beijing University of Aeronautics and Astronautics*.

[57] Aziz M. A. E., Ewees A. A., Hassanien A. E. (2017). Whale optimization algorithm and moth-flame optimization for multilevel thresholding image segmentation. *Expert Systems with Applications*.

[58] Upadhyay P., Chhabra J. K. (2020). Kapur’s entropy based optimal multilevel image segmentation using Crow Search Algorithm. *Applied Soft Computing*.

[59] Bao X., Jia H., Lang C. (2019). A novel hybrid Harris hawks optimization for color image multilevel thresholding segmentation. *IEEE Access*.

